RETRACTED

# Computed Tomography Image Characteristics before and after Interventional Treatment of Children's Lymphangioma under Artificial Intelligence Algorithm

**DOI:** 10.1155/2021/2673013

**Published:** 2021-12-09

**Authors:** Chuangao Yin, Song Wang, Deng Pan

**Affiliations:** Department of Image, Anhui Children's Hospital, Hefei, 230051 Anhui, China

## Abstract

The artificial intelligence algorithm was used to analyze the characteristics of computed tomography (CT) images before and after interventional treatment of children's lymphangioma. Retrospective analysis was performed, and 30 children with lymphangioma from the hospital were recruited as the study subjects. The ultrasound-guided bleomycin interventional therapy was adopted and applied to CT scanning through convolutional neural network (CNN). The CT imaging-related indicators before and after interventional therapy were detected, and feature analysis was performed. In addition, the CNN algorithm was adopted to segment the image of the tumor was clearer and more accurate. At the same time, the Dice similarity coefficient (DSC) of the CNN algorithm was 0.9, which had a higher degree of agreement. In terms of clinical symptoms, the cured children's lesions disappeared, the skin surface returned to normal color, and the treatment was smooth. In the two cases with effective treatment, the cystic mass at the lesion site was significantly smaller, and the nodules disappeared. CT images before interventional therapy showed that lymphangiomas in children were more common in the neck. The cystic masses at all lesion sites varied in diameter and size, and most of them were similar to round and irregular, with uniform density distribution. The boundary was clear, the cyst was solid, and there were different degrees of compression and spread to the surrounding structure. Most of them were polycystic, and a few of them were single cystic. After interventional treatment, CT images showed that 27 cases of cured children's lymphangioma completely disappeared. Lymphangioma was significantly reduced in two children with effective treatment. Edema around the tumor also decreased significantly. Patients who did not respond to the treatment received interventional treatment again, and the tumors disappeared completely on CT imaging. No recurrence or new occurrence was found in three-month follow-up. The total effective rate of interventional therapy for lymphangioma in children was 96.67%. The CNN algorithm can effectively compare the CT image features before and after interventional treatment for children's lymphangioma. It was suggested that the artificial intelligence algorithm-aided CT imaging examination was helpful to guide physicians in the accurate treatment of children's lymphangioma.

RETRACTED

## 1. Introduction

In the traditional diagnosis and treatment method, the clinician firstly makes an intentional diagnosis and then completes the diagnosis process through the cooperation of clinical symptom examination and analysis of various examination results [1]. Artificial intelligence is a technology that is defined to explore and develop how to simulate human intelligence through efficient and optimized means and to continuously expand and extend human intelligence [2]. This new type of technology on the one hand ensures patient's recognition of the accuracy of the imaging diagnosis results; on the other hand, it reduces the workload of the imaging doctors, allowing clinicians to judge the diagnosis and treatment results more quickly and accurately [3]. At present, medical artificial intelligence applications are mostly related to the diagnosis and detection of medical images, such as computed tomography (CT) imaging. The medical imaging artificial intelligence algorithm uses the default pixels of medical images to filter out effective image features, then learns and simulates clinicians' diagnosis and treatment techniques. The collected big data is subdivided according to the effective characteristics, and then, the reorganization and judgment are completed in turn, finally showing the diagnosis and treatment results with strong characteristics and high sensitivity [4]. Among them, the most widely used is convolutional neural networks (CNN). It delineates the area where the lesion occurred in the original CT scan image and then performs a series of subsequent quantitative and qualitative in-depth analysis of these areas. Scholars such as Masood et al. used artificial intelligence algorithms to compare and analyze the chest CT images collected from various databases. The results showed that after clinicians were assisted in diagnosis through the deep convolutional network algorithm, the diagnosis accuracy can reach an average of 85%, and the staging accuracy of lung cancer patients from T1 to T4 can reach up to 91% [5].

Lymphangioma in children is a benign tumor lesion in the lymphatic system caused by abnormal proliferation of endothelial cells on the lymphatic vessel wall [1]. Lymphangioma is a common disease in children. Congenital occurrence is mainly because the development of lymphatic vessels is not complete, and the innate lymphatic sac cannot normally drain to the middle smoke vein, so that the normal lymphatic structure that has been fully differentiated is abnormal, or the lymphatic structures that are not connected to the perfect drainage pathway and thus are shielded or the lymphocytic sac proliferates [6]. The acquired disease is mostly caused by lymphatic blockage, resulting in abnormal diameter of lymphatic vessels and cystic space malformations [7]. Lymphangiomas in children are usually classified into three types according to the diameter of the lesion, including cystic lymphoma, spongy lymphoma, and mixed lymphoma. This disease can occur in many parts of the body, but mainly in the head, neck, and face, accounting for about 75% of lymphangiomas in other parts [8]. Clinical manifestations also vary depending on the site and size of the lesion. Most of them grow as progressive painless masses, which affect the tissue structure around lymphatic vessels by means of compression and invasion. In the case of infection or secondary hemorrhage, the mass expands rapidly, resulting in serious complications such as obstruction of the airway [9]. At present, lymphangioma in children is usually diagnosed by puncture, which removes the lymphoid tissue and then carries out a follow-up routine examination. The treatment methods include surgery and sclerotherapy [10]. Clinical surgical resection is mainly aimed at some superficial lymphangiomas whose clinical symptoms are subcutaneous soft mass, smooth skin surface, and cystic touch but no pain. If the lymphangioma is located in the depth, there are no obvious clinical symptoms, so ultrasound and CT imaging assistance is needed [11]. Surgery can be complete resection of the lesion, but the surgical trauma is large, and postoperative recurrence is easy. The use of interventional therapy can solve the problem of large surgical trauma and easy recurrence. Studies have shown that the use of ultrasound interventional injection of bleomycin in the treatment of lymphatic malformations in the head and neck of infants and young children has found that the cure rate can reach 94.44% [12].

RETRACTED

The clinical manifestations and symptoms of lymphangioma in children are complex and diverse, and there are no specific clinical symptoms, so the early identification and diagnosis of this disease is difficult to a certain extent. At present, there are few data on the application of CNN in CT image processing of children's lymphangioma. Therefore, this article intended to use retrospective analysis to investigate the effect of CNN on CT imaging lesion segmentation of children with lymphangioma in children who had received ultrasound-guided interventional therapy for lymphangioma. The changes in CT imaging before and after treatment were analyzed to apply intelligent algorithms to assist in the diagnosis of children's lymphangioma and improve the efficiency of clinical diagnosis, aiming to provide a reference for analyzing the curative effect of interventional treatment of children's lymphangioma through CT imaging features.

## 2. Methods

### 2.1. Research Objects

A total of 30 children with lymphangioma admitted to the hospital from March 2018 to March 2020 were collected as the subjects of this study. There were 17 cases of boys and 13 cases of girls. The age ranged from three months to nine years old, with an average age of 55.56 ± 13.29 months. All 30 children were diagnosed as lymphangioma by surgical pathology. The course of the disease ranges from three months to three years. There were 21 cases of children with soft contact mass in the head and neck, chest, and abdomen, which tended to become larger. Nine children were admitted to hospital due to obvious abdominal symptoms, including lesions located in the mesentery, omentum majus, and retroperitoneum.

Inclusion criteria: (i) the age of patients ranged from three months to nine years; (ii) according to the 2020 CSCO Guidelines for Diagnosis and Treatment of Lymphoma in Children and Adolescents, the patient was clearly diagnosed as lymphangioma; (iii) all clinical data and information of the children were complete; (iv) the child was born normal without other congenital diseases; (v) preoperative CT scan was feasible.

Exclusion criteria: (i) children with autoimmune diseases, such as autoimmune hemolytic anemia; (ii) the child had hereditary coagulation dysfunction; (iii) patients with mental or consciousness disorders or poor compliance; (iv) patient with a history of surgical treatment.

All the families of the children in this study had signed the informed consent, and the study had been approved by the Ethics Committee of the hospital.

### 2.2. Interventional Treatment Methods

The interventional treatment method in this study was based on the *Guidelines for diagnosis and Treatment of Hemangioma and Vascular Malformations 2019* and was improved. As the surgical site involved great blood vessels and other parts, it was necessary to ensure the absolute silence of the child during the surgical process. The need for general anesthesia before surgery was determined based on child's age and adherence to the surgical treatment. All children had undergone skin tests for penicillin, which were negative. Bleomycin was injected under ultrasound guidance for interventional therapy, and the injection dose was 10 mg/m^2^ per body surface area according to the drug instructions. Ultrasound positioning was performed before injection and the color Doppler ultrasound machine was used. For the first injection, one-third of the drug was injected intramuscular first, and the child was closely observed. If no reaction occurred, the rest of the drug was injected again. The children were reviewed one-three months after surgery. If the disease still existed in the follow-up of diagnosis and treatment, it was necessary to continue to give treatment to the child and visit again.

RETRACTED

### 2.3. Scanning Methods

Before CT scan, all the 30 children were normal through routine laboratory examination. Upon admission, contrast-enhanced CT scans were performed to confirm the location, diameter, and characteristics of the cystic mass. The CT scanning instrument was 64 slice spiral CT scanner. The children were fasting for four hours before CT scan. The thickness of CT was set between 4 and 8 mm, iopromide 300 injection was used for enhanced imaging scanning, and the dose was calculated according to 2 mL/kg. High pressure syringe was injected through venous vessels, and dynamic multiphase CT scan was performed with the scanning time set to 0.9 s. After the scan, all raw data was transferred to the workstation. If the child did not cooperate during CT scan, chloral hydrate should be used to help sedation of the child at a dose controlled below 1 mg/kg. Both the original image obtained from the scan and the processed image should be evaluated by at least two professional imaging physicians. In case of disagreement, a final agreement should be reached through negotiation.

### 2.4. CT Image Processing Flow Based on CNN Algorithm

CNN algorithm directly takes the original data image of CT image as input data and then obtains data features with considerable weight through analysis. It can make the important feature extraction work of traditional identification algorithm less complicated. The network structure flowchart of CNN is shown in Figure 1.

### 2.5. Evaluation Index Based on CNN Algorithm

To apply the CNN algorithm to CT images accurately, a main indicator is first used to evaluate the results of the CNN algorithm. The similarity coefficient (DSC) refers to the degree of agreement between the correctly divided data in the CT image result and the original lesion. The higher the degree of agreement, the more accurate the division result of the CNN algorithm. The calculation method is as follows.

(1) $$\begin{array}{c} \text{DSC}=\frac{2\;|\;A\cap B\;|\;}{\;|\;A\;|\;+\;|\;B\;|\;}\times 100\%. \end{array}$$

In the above equation, *A* represents the data result of the division of the tumor by the clinician, while *B* represents the result of the division of the tumor by the CNN algorithm. *A*∩*B* represents the consistent result of *A* and *B*. Canny algorithm [13] is introduced for comparison in terms of DSC.

### 2.6. Treatment Evaluation Indexes

All children were classified by this index to indicate the treatment effect. Cure: after imaging and routine examinations, it was found that the lesion disappeared, and there was no mass. Effective: after the child was treated, it was found that the tumor size of the lesion became smaller, and the clinical symptoms were alleviated, but the degree of improvement was less than 60%. Ineffective: after interventional treatment, it was found that the tumor did not shrink or showed a tendency to become larger.

RETRACTED

### 2.7. Image Result Analysis Indexes

After CT scan, the clinical general data and surgical pathological examination data were combined. The site, diameter, shape, density, structure, and image characteristics of lymphangioma were analyzed.

## 3. Results

### 3.1. Results of Gender and Age Distribution of All Children with Lymphangioma

The information of sex and age of 30 children were obtained from the retrieval system of medical record management department.  Table 1 showed the specific results.

### 3.2. CNN Algorithm Processing Results of CT Images

After CT images were analyzed and processed with CNN algorithm, the following partition results were obtained. According to Figure 2, the image of tumor segmentation by CNN algorithm was clear and accurate.  Figure 2(a) represented the original CT image of a lymphangioma.  Figure 2(b) represented clinician's classification of tumor lesions.  Figure 2(c) represented the segmentation results of tumor using CNN algorithm.  Figure 2(d) represented the image of tumor lesions divided by Canny algorithm.

### 3.3. CNN Algorithm Evaluation Index Results

DSC was used to evaluate the performance of CNN algorithm applied in CT images. It was found that the DSC of the CNN algorithm was 0.90, while the DSC of the Canny algorithm was reported to be 0.85. It showed that the CNN algorithm used in this research was obviously higher than the Havaei algorithm DSC, and the agreement was better (Figure 3).

### 3.4. CT Image Analysis

The location of the lesion was as follows. There were 30 children with lymphangioma, of which 15 children with the disease on the neck and 6 children with the parotid gland. There were four children located on the cheeks, two children located under the armpits, two children located on the abdomen, and 1 child located on the front chest. Lymphangioma in children mainly occurred in the head and neck. In Figure 4, (a) represented the image of cervical lymphangioma, (b) represented the image of parotid lymphangioma, (c) represented the image of cheek lymphangioma, (d) represented the image of axillary lymphangioma, (e) represented the image of abdominal lymphangioma, and (f) represented the image of anterior thoracic lymphangioma.  Table 2 and Figure 4 showed the details.

- Diameter. After inspection, the diameter of cystic masses in all lesions was different. The diameter of the mass was calculated by taking the largest cross-sectional area measured. The diameter of the largest mass was 13.7 cm × 10.3 cm, and the diameter of the smallest mass was 2.4 cm × 3.1 cm
- Morphology and density. Most of the lymphangiomas in the scan image were similar to circular and irregular, and the density distribution was relatively uniform. The boundary was clear, the cyst was solid, and there were different degrees of compression and spread to the surrounding structure
- Types of lesions. According to the results of all children, lymphangiomas were mostly polycystic, and a few were single cystic. Among them, there were 27 cases of polycystic type and 3 cases of single cystic type. In Figure 5, (a) was polycystic lymphangioma, and (b) was mono cystic lymphangioma. Figure 5 showed the details

RETRACTED

### 3.5. CT Examination after Treatment

All children underwent CT scan again after interventional treatment. It was found that in the CT images of 27 cured children, the lymphangioma disappeared completely. In the CT images of two children with effective treatment, the lymphangioma was significantly reduced, and the edema around the tumor was also significantly reduced. CT imaging examination of a child who was ineffective in treatment revealed a wide range of lesions. After reexamination and follow-up, after receiving interventional treatment again, children's tumor disappeared after CT imaging examination. No recurrence or new disease was found in the three groups of children during the three-month follow-up.

### 3.6. Evaluation of Treatment Efficacy

Through the treatment results of 30 children, it was found that 27 cases were cured, 2 cases were effective in treatment, and 1 case was ineffective in treatment. The total effective rate of treatment was 96.67% (29/30). Among them, the two children with effective treatment were children with lymphangioma located in the neck, and the one with no treatment was children with lymphangioma located in the abdomen. The swelling at the diseased part of the cured child disappeared, the skin surface returned to normal color, and the treatment was smooth and level. The cystic masses in the lesions of the two children with effective treatments became smaller, and the nodules disappeared. There was no significant change in the lesions of the children who had ineffective treatment results (as shown in Figure 6).

## 4. Discussion

Lymphangioma is a kind of benign angioma located in the lymphatic system, which occurs frequently in congenital. It is most common in children and minors, and more than 90% of cases occur between infants and two years old [14]. The incidence of lymphangioma is only second to hemangioma, ranking the second among angiomas [15]. Lymphangioma occurs in the mesoderm, mainly due to the abnormal development of primitive lymphatic vessels or abnormal proliferation of lymphatic endothelial cells [16]. Lymphangiomas can occur anywhere on the body with the lymphatic system, but clinical studies found that the main site is the head and neck. Secondly, it was found in axilla, parotid gland, face, mediastinum, oral cavity, and other parts [17]. It was found that among the 30 cases of children with lymphangioma, the lesion was located in the neck in 15 cases, accounting for the general proportion. Six cases were located in parotid gland, accounting for 20%. Four cases were located in cheek, accounting for 13.3%. Two cases were located in the armpit, accounting for 6.7%. There were two cases with abdominal location, accounting for 6.7%. This was consistent with the reported research results [18]. At present, the clinical features of lymphangioma vary according to the location and size of the tumor lesions [19]. Traditionally, lymphangioma is treated by surgical resection of the tumor, but it is difficult to complete surgical resection of the tumor, and the postoperative recurrence rate is high, up to about 55%. In addition, there are also many complications [20]. Therefore, many patients receive interventional therapy as an alternative to surgical removal of lymphangioma. On the one hand, interventional therapy can keep the skin structure and soft tissues intact during the treatment process; on the other hand, it will not cause serious complications. In this study, 30 children were treated with ultrasound-guided injection of bleomycin, and no comorbidities were found. In 27 cases of cured children, the tumor disappeared, the skin surface returned to normal color, and the treatment was smooth and smooth. In two patients with effective treatment, the cystic mass was significantly smaller, and the nodules disappeared. None of the children had serious complications. This was consistent with research reports.

RETRACTED

Artificial intelligence algorithm is an emerging technology that uses computer algorithms to learn and simulate human thinking and abilities. Guo et al. (2019) [21] stated that artificial intelligence technology has not only been used in the differential diagnosis and prognostic evaluation of diseases but also in clinical data analysis and imaging diagnosis to analyze the medical imaging results obtained, so as to obtain accurate medical information. Lesion division of medical images plays an important role in the effective processing of images using algorithms in the clinic. It can extract the scope of the lesion and conduct qualitative and quantitative in-depth analysis, which plays an important role in medical diagnosis and identification [22]. The combination of CNN algorithm and CT image was adopted to segment the tumor lesions of children with lymphangioma, and the effect was compared with that of Canny algorithm. It was found that the image map of the tumor body segmentation using the CNN algorithm was relatively clearer and more accurate. The CNN algorithm was obviously higher than the reported algorithm DSC, and the agreement was better. It was suggested that the CNN algorithm was of more clinical application value for CT image segmentation of lesions.

Based on the above analysis, the results suggested that the CNN algorithm segmented the image of children's lymphangioma tumors with clearer and more accurate range. The CNN algorithm DSC was 0.9, which was obviously higher than the reported algorithm DSC and had a better agreement.

CT imaging before interventional treatment revealed that CT images showed that 15 children with lymphangioma lesions located in the neck, indicating that lymphangioma in children was more likely to occur in the neck. The diameters of cystic masses at all lesions varied in size, and most of the lymphangiomas were similar to round and irregular. The density distribution was relatively uniform, the boundary was clear, the capsule was solid, and the surrounding structure had different degrees of compression and spreading morphological distribution. Lymphangiomas were mostly multicystic, and a few were single cystic.

In terms of the clinical symptoms after the interventional treatment, the lumps in the diseased part of the cured child disappeared, and the skin surface returned to normal color, smooth, and level. The cystic mass at the affected part of the child with effective treatment was significantly smaller, and the nodules disappeared. CT imaging revealed that the lymphangiomas of 27 cured children disappeared completely, and the lymphangiomas of 2 children with effective treatment decreased significantly. The edema around the tumor also decreased significantly. After the children who did not respond to the treatment received interventional therapy again, the tumors on CT imaging also disappeared completely. In addition, no recurrence or new disease was found in the three groups of children during the three-month follow-up. The total effective rate of interventional therapy for childhood lymphangioma was 96.67% (29/30).

## 5. Conclusion

This study used a CNN algorithm to segment the CT images of children's lymphangiomas. The results proved that the algorithm can perform more accurate segmentation and provide more auxiliary forms for imaging doctors in the diagnosis and treatment of children's lymphangiomas. The imaging changes of children with lymphangioma before and after interventional treatment were obtained through CT image feature analysis, which showed that CT image feature analysis can be used as a method for judging the clinical treatment results of children with lymphangioma, providing a reference for the clinical treatment effect. However, there were few research subjects included in this study, and the contrast of different pathological types of childhood lymphangioma was not strong enough. Therefore, more samples and different pathological types were needed to conduct research in the future.

RETRACTED

## Figures and Tables

**Figure 1:** Flow chart of CNN network structure.

**Figure 2:** CNN algorithm for CT image processing. (a) represented the original CT image of lymphangioma; (b) represented clinician's classification of tumor lesions; (c) represented the result of tumor classification using the CNN algorithm; and (d) represented the algorithm that has been reported to use the algorithm to divide tumor lesions picture.

**Figure 3:** DSC comparison of the two algorithms.

**Figure 4:** CT images of the distribution of each part of the lesions. ((a) image of cervical lymphangioma; (b) image of parotid lymphangioma; (c) image of cheek lymphangioma; (d) image of axillary lymphangioma; (e) image of abdominal lymphangioma; (f) image of anterior chest lymphangioma).

**Figure 5:** Two different types of lesions ((a) polycystic lymphangioma; (b) mono cystic lymphangioma).

**Figure 6:** Proportion of treatment assessment results of children (%).

**Table 1:** Age and sex of the children.

Sex	Age (years old)	Number of cases	Total
Male	<5	10	17
	≥5	7	
Female	<5	8	13
	≥5	5	

**Table 2:** Distribution of lesions in children.

Classification	Neck	Parotid gland	Cheek	Armpit	Abdomen	Front chest
Number of children (cases)	15	6	4	2	2	1
Proportion (%)	50	20	13.3	6.7	6.7	3.3

## Data Availability

The data used to support the findings of this study are available from the corresponding author upon request.
